# Congenital Granular Cell Epulis in a Newborn: Diagnostic and Surgical Challenges in a Resource‐Limited Setting—A Case Report

**DOI:** 10.1002/ccr3.72524

**Published:** 2026-04-26

**Authors:** Abdisalam Ismail Hassan, Aweis Abdullahi Sheikh, Balqiz Mohamed Kulle, Eid Mohamed Jama, Fardowso Ali Mohamud, Ahmed Muhammad Bashir

**Affiliations:** ^1^ Faculty of Medicine and Health Sciences Jamhuriya University of Science and Technology Mogadishu Somalia; ^2^ Pathology Department Mogadishu Somali–Türkiye Recep Tayyip Erdoğan Training and Research Hospital Mogadishu Somalia; ^3^ Anesthesia and Critical Care Department Mogadishu Somali–Türkiye Recep Tayyip Erdoğan Training and Research Hospital Mogadishu Somalia; ^4^ Internal Medicine Department Somali Sudanese Specialized Hospital Mogadishu Somalia

**Keywords:** case report, congenital epulis, congenital granular cell epulis, neonatal tumor, newborn oral mass, resource‐limited setting, Somalia

## Abstract

Congenital granular cell epulis (CGCE) is a rare benign tumor of the neonatal gingiva, with fewer than 250 cases reported worldwide. It presents most commonly as a pedunculated mass arising from the maxillary alveolar ridge and may interfere with feeding or, rarely, respiration. Early recognition is essential, particularly in resource‐limited settings where diagnostic tools may be restricted. We report the case of a 7‐day‐old female neonate born at term with a 2 × 1.5 cm smooth, pedunculated intraoral mass originating from the anterior maxillary alveolar ridge. The lesion did not impair respiration or feeding. Baseline laboratory investigations were normal, and the mass was electively excised under general anesthesia on day 7 of life. Histopathology revealed large polygonal cells with granular eosinophilic cytoplasm and atrophic overlying epithelium, confirming the diagnosis of congenital granular cell epulis. Immunohistochemical studies were not available. Postoperative recovery was uneventful, with complete resolution and no recurrence at the one‐month follow‐up. CGCE can be effectively managed with simple surgical excision, even in low‐resource environments. Increased awareness among clinicians is essential to ensure timely diagnosis and avoid unnecessary interventions.

## Key Clinical Message

Congenital granular cell epulis is a rare benign neonatal gingival tumor that may mimic other oral masses. Early clinical recognition and simple surgical excision result in excellent outcomes. This case demonstrates that accurate diagnosis and effective management are achievable even in resource‐limited settings without advanced diagnostic tools such as immunohistochemistry.

## 1 Introduction

Congenital epulis, also known as granular cell tumor of the gingiva, congenital granular cell tumor, congenital granular cell fibroblastoma, congenital granular cell myoblastoma, Neumann's tumor, and congenital granular epulis, is a rare benign lesion of the gingiva [1]. A marked female preponderance has been reported, with an incidence estimated as low as 0.0006% [2]. Fewer than 250 cases of congenital granular cell epulis (CGCE) have been documented in the literature [3]. CGCE shows a striking female predominance, with a reported female‐to‐male ratio of approximately 8–10:1 [4]. Clinically, the lesion typically presents as a smooth‐surfaced, lobular, sessile, or pedunculated swelling. Larger lesions may interfere with respiration and feeding owing to their intraoral origin [5]. When large, these lesions may compromise breastfeeding and, less commonly, respiration, underscoring the need for timely evaluation at birth [4, 6]. Although histologically benign, congenital epulis can result in neonatal asphyxia or feeding difficulties, necessitating prompt intervention [7].

In most cases, diagnosis relies primarily on clinical presentation and classical histopathological features, making clinician awareness essential to prevent misdiagnosis and inappropriate management. Reporting cases from diverse geographic regions is therefore crucial for improving global epidemiological understanding and guiding diagnostic and surgical strategies, particularly in environments with limited diagnostic resources.

We present the first documented case of CGCE in Somalia, detailing the clinical presentation, surgical management, and histopathological findings. This case highlights key diagnostic considerations and the challenges of managing rare neonatal tumors in resource‐limited settings and contributes valuable regional data to the global literature.

## 2 Case History and Examination

A 7‐day‐old female neonate weighing 3585 g was born at our hospital to a 29‐year‐old mother (G3P3) from a non‐consanguineous marriage. The pregnancy and delivery were uneventful, and the infant was delivered at term via spontaneous vaginal delivery with no reported maternal illnesses, medication exposure, or perinatal complications.

At birth, a firm, pedunculated, smooth‐surfaced pink mass was observed protruding from the oral cavity, originating from the anterior maxillary alveolar ridge (Figure 1). The lesion measured approximately 2 × 1.5 cm, was non‐ulcerated, and did not bleed on gentle manipulation. The mass did not cause respiratory distress or interfere with feeding, and the neonate was able to breastfeed adequately.

**FIGURE 1:** Clinical photograph showing a congenital granular cell epulis prior to surgical excision.

On examination, the infant appeared active and well‐perfused with normal vital signs for age. Chest auscultation was clear bilaterally, heart sounds were normal without murmurs, and the abdomen was soft and non‐distended. Neurological examination demonstrated normal tone and appropriate neonatal reflexes. Oropharyngeal examination revealed a solitary pedunculated mass arising from the anterior maxillary alveolar ridge with intact mucosa and no signs of infection or airway obstruction. No additional congenital anomalies were identified.

## 3 Differential Diagnosis, Investigations, and Treatment

The differential diagnoses considered included congenital granular cell epulis, congenital epulis, hemangioma, fibroma, and teratoma. Baseline laboratory investigations—including complete blood count, C‐reactive protein, serum electrolytes, liver and renal function tests, and coagulation profile—were within normal limits, confirming the infant's suitability for surgery.

The mass was surgically excised under general anesthesia on day 7 of life. A simple pedicle excision was performed with minimal bleeding while preserving the underlying alveolar ridge. Postoperative recovery was uneventful, and no residual lesion or deformity was noted immediately after excision (Figure 2). The infant tolerated the procedure well, resumed oral feeding within a few hours, and was discharged on postoperative day 2 in stable condition.

**FIGURE 2:** Postoperative appearance following surgical excision of congenital granular cell epulis.

## 4 Conclusion and Results (Outcome and Follow‐up)

Histopathological examination demonstrated a submucosal proliferation of large polygonal cells with abundant eosinophilic granular cytoplasm and small central nuclei (Figure 3A,B). The overlying squamous epithelium appeared atrophic, likely due to pressure from the underlying mass. These findings confirmed the diagnosis of congenital granular cell epulis, a rare benign tumor of the neonatal gingiva.

**FIGURE 3:** (A) High‐magnification image showing proliferation of large cells with granular cytoplasm. (B) H&E‐stained section showing squamous epithelium and underlying granular cytoplasm.

At the one‐month follow‐up, the infant showed complete healing with normal feeding and no evidence of recurrence.

## 5 Discussion

CGCE is an uncommon benign tumor of the neonatal oral cavity, with fewer than 250 cases reported in the literature [3]. Its pathogenesis remains uncertain, with several theories proposed, including myoblastic, neurogenic, odontogenic, fibroblastic, histiocytic, and endocrinologic origins [8].

The lesion has been described under various terms, including congenital epulis and Neumann's tumor. The World Health Organization standardized the terminology as “congenital granular cell epulis,” which was adopted in this report [9].

CGCE most frequently arises from the maxillary alveolar ridge, occurring approximately three times more often than in the mandible [3, 9]. Most cases present as solitary lesions, although multiple lesions have been reported in a minority of patients. The clinical features observed in our patient are consistent with these findings.

Prenatal detection may be possible during the third trimester using ultrasound or fetal MRI; however, many cases are identified at birth. A strong female predominance has been consistently reported [10], which aligns with our case. Despite this observation, no definitive hormonal association has been established [11].

Typically, CGCE presents as a painless lesion that does not increase in size after birth and maintains a consistent appearance [12]. Management depends on the presence of functional impairment. Surgical excision is recommended when feeding or airway compromise is suspected [13]. In our patient, elective excision was successfully performed, with no postoperative complications or recurrence.

Immunohistochemistry may assist in differentiating CGCE from other granular cell lesions, particularly adult granular cell tumors, which are usually S100‐positive. In contrast, CGCE is typically S100‐negative and may express vimentin and CD68. In this case, IHC was not performed due to limited resources. However, the diagnosis was confidently established based on classical histopathological features, consistent with previously reported cases.

This report contributes additional clinical data from Somalia and highlights that accurate diagnosis and effective management can be achieved through careful clinical and histopathological evaluation, even in settings with limited diagnostic capabilities.

## 6 Conclusion

CGCE is a rare benign neonatal tumor with an excellent prognosis following surgical excision. Early recognition is essential to prevent potential feeding or airway complications. This case illustrates that effective diagnosis and treatment are achievable using standard clinical and histopathological approaches, even in low‐resource healthcare environments.

## Author Contributions

**Abdisalam Ismail Hassan:** conceptualization, data curation, resources, writing – original draft. **Aweis Abdullahi Sheikh:** data curation, methodology, resources. **Balqiz Mohamed Kulle:** conceptualization, writing – original draft. **Eid Mohamed Jama:** data curation, methodology, writing – original draft. **Fardowso Ali Mohamud:** data curation, methodology, writing – original draft. **Ahmed Muhammad Bashir:** supervision, writing – review and editing.

## Funding

The authors have nothing to report.

## Ethics Statement

In our institute, ethical approval is not required for the publication of case reports, so our hospital is waived for case reports, and informed written consent was obtained from the patient's legal guardian for using their information and publishing the case report, provided that identifying data remains anonymous.

## Consent

Written informed consent was obtained from the patient's legal guardian for publication, ensuring anonymity.

## Conflicts of Interest

The authors declare no conflicts of interest.

## Data Availability

All relevant data supporting the findings of this case report are included within the article. Additional details are available from the corresponding author on reasonable request.
